The article "Correlation between Vaginal Microecological Status and Prognosis of CIN Patients with High-Risk HPV Infection" was published in 2022. Journal: Biomed Res Int.

# Correlation between Vaginal Microecological Status and Prognosis of CIN Patients with High-Risk HPV Infection

**DOI:** 10.1155/2022/3620232

**Published:** 2022-04-14

**Authors:** Huizhen Zhang, Shuangling Jin, Aifang Ji, Chunyan Zhang, Shujing Shi

**Affiliations:** ^1^Department of Gynecology, Heping Hospital, Changzhi Medical College, Changzhi 046000, China; ^2^Department of Laboratory Medicine, Heping Hospital, Changzhi Medical College, Changzhi 046000, China

## Abstract

Many microorganisms live in the vagina of healthy women. They interact with and compete with the microenvironment in the female vagina to form a dynamic balance of the microenvironment in the female vagina. However, imbalanced vaginal microecology can lead to vaginal resistance to pathogenic microorganisms. Poor capacity can cause women to develop infections of the reproductive tract. This article analyzes the vaginal microecological status of women with high-risk HPV infection for more than 6 months and healthy women and explores the risk factors that cause long-term high-risk HPV infection for timely detection and regulation of possible vaginal microecological imbalance in women with high-risk HPV infection for more than 6 months to prevent further development of cervical lesions in such patients. This article covers women with a sexual life history who attended the gynecology department of a hospital from January 2020 to September 2021. There were 280 patients in the experimental group: positive high-risk HPV; and there were 140 patients in the control group: negative high-risk HPV test. The correlation between vaginal microecology of CIN patients and patient prognosis according to the subject's vaginal microecology test results and prognosis of various levels of cervical lesions was analyzed. The experiment proved that the detection rate of normal vaginal microecology in the experimental group was 12.14% (34/280) compared with the detection rate of 29.29% (41/140) in the control group, and there was a trend of decrease, and the difference was statistically significant (*χ*^2^ = 17.23, *P* < 0.05). The detection rate of vaginal BV in the experimental group was 10.36% (29/280) compared with the detection rate of 5.0% (7/140) in the control group, and the difference was statistically significant (*χ*^2^ = 5.19, *P* < 0.05). This indicates that women with high-risk HPV infections for 6 months or longer have a higher incidence of vaginal microecological imbalances than healthy individuals and aggressive vaginal microecological screening. It is necessary to carry out the program. Detect and treat possible abnormal conditions in time to prevent the further onset of the disease.

The article "Correlation between Vaginal Microecological Status and Prognosis of CIN Patients with High-Risk HPV Infection" was published in 2022. Journal: Biomed Res Int.

## 1. Introduction

HPV is the main pathogenic factor of cervical cancer. Studying its carcinogenic mechanism and factors affecting the occurrence and development of cervical cancer plays an important role in the prevention and treatment of cervical cancer. Multiple HPV infections can increase the risk of cervical lesions in patients, accelerate the progression of cervical lesions, and affect the sensitivity of cervical cancer patients to treatment and affect the prognosis of patients. This effect is associated with accelerated HPV recombination during multiple HPV infections, the formation of new types of HPV with greater pathogenicity and invasiveness, faster disease progression, and increased disease malignancy. Therefore, it is of particular importance to study the correlation between the various clinical features of cervical lesions caused by multiple HPV infections and whether multiple HPV infections promote HPV recombination and its mechanism.

High-risk HPV infections are mainly transmitted through sex. Cervicitis and CIN caused by infection are the most common cervical problems in clinical practice. If they are not treated in time, they may progress to cervical malignant tumors. Although the health departments around the world attach great importance to high-risk HPV infection and invest a lot of resources in the prevention, screening, and vaccine development of high-risk HPV, the detection rate and mortality of cervical cancer are still on the rise. The virus in most infected people does not last for more than 6 months. Most women can quickly get rid of high-risk HPV by relying on the self-cleansing capacity of the vaginal microecosystem and the self-repair of cervical epithelial cells. However, some women are still unable to get rid of high-risk HPV infections in their bodies. The continued action of high-risk HPV ultimately leads to the development of CIN and cancer.

The cervix is always surrounded by the vaginal microecological environment. The cervix and vagina infected with high-risk HPV are inextricably linked to the vaginal microecological environment. Whether there is a clear difference between the vaginal microecological status of people with high-risk HPV long-term infection and healthy people, domestic and foreign scholars have not yet reached a consensus. In order to assess the vaginal microecological status of high-risk HPV infection cervical intraepithelial neoplasia, 241 high-risk HPV-infected CIN patients diagnosed and treated by the Cervical Disease Center were selected as the experimental group, and 168 women who underwent physical examination in the outpatient clinic were studied. The HPV-negative and normal cytological examination results were used as a control group to compare the differences in the vaginal microecological status between the two groups. However, the lack of experimental data in his study led to small differences in the sample set, resulting in inaccurate results [1]. There is an indirect connection between multiple sex partners (MSP) and cervical intraepithelial neoplasia (CIN) and even cervical cancer (CC). MSP can also cause bacterial vaginosis (BV). The relationship between MSP, BV, human papillomavirus (HPV) infection, and CIN/CC development in Chinese women remains unclear. Rabaan et al. retrospectively analyzed 549 female patients who had been to the physical examination center. MSP information was obtained, and vaginal microecology, HPV, and cervical conization pathology (CCP) tests were performed when necessary. In patients with different severity of BV, MSP status is different. In addition, as the severity of BV increases, the HPV-positive rate increases. At the same time, MSP is significantly related to HPV-positive results, including HPV16, HPV18, and other high-risk HPV infections. The percentage of positive CCP results in the MSP group was significantly higher. Similarly, higher severity of BV means that CIN/CC is progressing more severely. However, its overall study lacks data support, and more data is needed to support its conclusions [2]. Pan et al. investigated the role of HPV16 DNA integration in cervical lesions in Han and Uyghur women and explored the relationship between virus integration and high cervical cancer incidence and low HPV infection rates. DNA was extracted from cervical lesion biopsy specimens of 379 Uyghur and 464 Han patients, and multiple quantitative polymerase chain reaction (qPCR) analyses were performed to determine the copy numbers of HPV16E2 and E6 genes. The copy number of HPV16DNA was evaluated based on the E2/E6 ratio. Among these cases, 122 Uyghur and 121 Han specimens were found to be HPV16-positive. In these two populations, the percentage of HPV16 integrated cases increased with the degree of cervical lesions (*P* < 0.05), but the testing equipment was immature at the time of the study, resulting in insufficient accuracy [3].

The article "Correlation between Vaginal Microecological Status and Prognosis of CIN Patients with High-Risk HPV Infection" was published in 2022. Journal: Biomed Res Int.

In the past, clinical studies on patients with high-risk HPV infections mostly focused on the relationship between HPV infection and simple vaginal inflammation. Few studies were conducted on the overall status of vaginal microecology in women with high-risk HPV infections over 6 months. This article focuses on the relationship between HPV multiple infections in cervical cancer patients and the clinical manifestations of cervical cancer, revealing the effects of multiple HPV infections on the clinical features of cervical cancer. By investigating the mechanism of this effect and discovering and controlling potential imbalances in the vaginal microeconomics in time, further development of cervical lesions and multiple HPVs in the future can be prevented. It may provide a more theoretical basis for the prevention, evaluation, and follow-up of patients with infectious diseases.

## 2. Correlation between High-Risk HPV Infection and Patient Prognosis

### 2.1. Vaginal Microecological Status of CIN Patients with High-Risk HPV Infection

#### 2.1.1. High-Risk HPV Infection and Normal Vaginal Microbiota

It is generally believed that a healthy vaginal microecological status is the following: the density of the colonizing bacteria in the vagina is between level II and level III, the diversity of the flora is between level II and level III, and lactobacilli occupy an absolutely dominant position in terms of quantity. No infection of pathogenic microorganisms such as BV, candidal vaginitis (VVC), and trichomonal vaginitis (TV) was found in the vagina, the number of white blood cells is less than 10/high-powered field of view, the pH value in the vagina is ≤4.5, which reflects that lactic acid Bacillus functions are positive for hydrogen peroxide; sialidase, which reflects BV infection; leukocyte esterase, which reflects the massive destruction of vaginal white blood cells due to inflammation; *β*-glucuronidase, which reflects the overgrowth of aerobic bacteria in the vagina and indicates possible VVC infection; or TV acetylglucosaminidase, etc., which are all negative. A healthy vaginal microecological environment has a protective function for the human body [4, 5], and an unbalanced vaginal microecological environment can easily cause the female reproductive tract to be attacked by various pathogens. Pathogens that invade the female reproductive tract can further aggravate the imbalance of vaginal microecology and form a vicious circle.

#### 2.1.2. High-Risk HPV Infection and Vaginal Lactobacillus and pH Value

Lactobacillus is the dominant bacteria that colonize the vagina of healthy women, and it is also the main force to maintain the vaginal microecological balance. It accounts for more than 95% of the total vaginal microbes, and 80 to 90% of women can isolate the bacteria in the vagina. The decrease in the number of lactobacilli reduces the resistance of the vagina to pathogenic microorganisms, resulting in the persistence of high-risk HPV infections. The specific mechanism of action still needs more in-depth research [6, 7]. It is ideal for women's vagina to maintain a pH value between 3.8 and 4.5. This acidic environment has a strong killing effect on most pathogens that invade the vagina. When internal or external changes cause the vaginal microecological balance to be disrupted, it will lead to changes in the vaginal pH value, and the abnormal pH value will aggravate the imbalance of the vaginal microecology, forming a vicious circle [8].

The article "Correlation between Vaginal Microecological Status and Prognosis of CIN Patients with High-Risk HPV Infection" was published in 2022. Journal: Biomed Res Int.

#### 2.1.3. Current Status of Clinical Application of Vaginal Microecological Testing

The concept of vaginal microecology was first proposed by the Obstetrics and Gynecology Infectious Diseases Cooperation Group of the Chinese Medical Association of our country and has been popularized and used for more than 10 years. Traditional vaginal secretion testing methods can only diagnose vaginitis with a clear pathogenic infection and are limited by the time of specimen collection, the quality of specimens, and the inspector's testing experience. The accuracy of the test results is not high, and the efficiency is low. In recent years, the female vaginal microecological detection system has the advantages of fast, simple, multiple results, clear morphological staining, comprehensive functional detection, etc., and the detection rate of pathogenic microorganisms is higher than that of traditional microscope detection methods, and it can be combined with the morphological and functional characteristics of the test samples to obtain more accurate and comprehensive inspection results [6, 9]. The application of the vaginal microecological assessment system, on the one hand, modifies the concept of reproductive tract infections, which diagnoses “vaginal disease” only after the discovery of pathogenic microorganisms. On the other hand, it goes beyond the existing concept of treating vaginal infections. It kills pathogens. The main purpose of improving diagnosis and treatment is to increase beneficial bacteria in the vagina and restore a healthy microecological condition of the vagina as a standard new concept that is a major advance in the diagnosis and treatment of vaginal infections. Therefore, if we want to fully understand the interaction between HPV infection and the human body, we need to use the accuracy and comprehensiveness of the vaginal microecological testing system to compare and analyze the vaginal microecological status of high-risk HPV-infected persons and healthy people [10, 11].

### 2.2. Artificial Neural Networks

#### 2.2.1. Single Neuron

In order to imitate the working mechanism of biological nerve cells, scientists have designed artificial neurons. Assuming that a neuron has three input data *x*_1_, *x*_2_, *x*_3_, the intensity of the neuron's action can be expressed as *w*_1_, *w*_2_, *w*_3_ by weight, plus a bias term *b*, which is sent into the cell for processing together [12, 13]. Thus, the input value of the neuron can be

(1) $$\begin{array}{c} \overset{3}{\underset{i=1}{\sum }}w_{i}x_{i}. \end{array}$$

The output value can be expressed as

(2) $$\begin{array}{c} Z=f\left(\overset{3}{\underset{i=1}{\sum }}w_{i}x_{i}+b\right). \end{array}$$

The symbol *f* represents the neuron function. According to the difference in solving the problem, the activation function is usually different; otherwise, it will affect the convergence of the algorithm. The commonly used activation functions are as follows, one is the Sigmoid activation function, the other is the Tanh activation function, the third is the ReLU activation function, and the fourth is the Maxout activation function. The mathematical formulas of Sigmoid function and Tanh function are shown in

(3) $$\begin{array}{c} f\left(h\right)=\frac{1}{1+e^{\left(-h\right)}},\\ f\left(h\right)=\tanh\left(h\right)=\frac{e^{h}-e^{-h}}{e^{h}+e^{-h}}. \end{array}$$

There are many similarities between the Sigmoid curve and the Tanh curve: Regardless of whether the input value is large or small, the Sigmoid function can control the value between 0 and 1; for extremely large negative numbers, the output value is 0, and for extremely large positive numbers, the output value is 1. Tanh is derived from Sigmoid, and its output value is between -1 and 1, with an average value of 0 [14, 15]. The calculation of the ReLU function is relatively simple: when the input value is less than 0, the output is 0; when the input value is greater than 0, the output is equal to the input. The formula is as follows:

(4) $$\begin{array}{c} f\left(h\right)=\max\left(0,h\right). \end{array}$$

The advantage of this activation function is that it can process data quickly and only needs to set a threshold. However, the ReLU function also has a relatively large drawback—the ReLU neuron processes large gradients and updates the parameters, which may easily cause the neuron to not activate the data [16]. The core idea of Maxout calculation is to take the maximum value of the corresponding position of the feature map of the previous layer as the output of the Maxout unit. The formula is shown in formula (5), where *k* is the number of feature maps output by Maxout:

(5) $$\begin{array}{c} \left\{\begin{array}{c} f_{i}\left(h\right)=\max\left(Z_{ij}\right),\;j\in \left[1,k\right],\\ Z_{ij}=h^{T}w_{ij}+b_{ij}. \end{array}\right. \end{array}$$

Maxout does not have a fixed curve and can fit any convex function, so the fitting ability is relatively good, and it contains the advantages of the ReLU function while avoiding its defects. Other activation functions include threshold functions and linear functions. Different functions have different characteristics, which constitute a neural network with different functions nowadays [17, 18].

The article "Correlation between Vaginal Microecological Status and Prognosis of CIN Patients with High-Risk HPV Infection" was published in 2022. Journal: Biomed Res Int.

#### 2.2.2. Neural Network

Similar to brain tissue being composed of countless nerve cells, ANN is also composed of many artificial neurons.  Figure 1 is a typical feedforward neural network. The small circle in the figure represents a neural processing unit, and some neurons form a layer of the network [19, 20]. The order of each layer is determined according to the sequence of information transmission. For example, the third layer only accepts the information output by the second layer. There is no feedback signal between each neural processing unit, and there is no feedback information between layers.

The input layer of a feedforward neural network structure contains multiple input neural nodes that represent the input values, and the input layer transfers data to the hidden layer for further processing. The processed values of the hidden layer cannot be directly observed during the operation of the neural network. The neuron has multiple inputs, but there is only one output value that can be sent to multiple neurons as input [21, 22]. The last layer is the output layer, which can have one or more output nodes. Multioutput neural networks can be applied to issues such as multiple results, such as computer performance evaluation. The input data of the network can use various computer hardware configurations. After processing, the output has either high performance, medium performance, or low performance. Suppose a forward neural network contains 3 network layers, the first layer is the input layer, the second layer is the hidden layer, and the third layer is the output layer. The input layer has 3 values {*x*_1_, *x*_2_, *x*_3_}, the weights corresponding to the hidden layer are {*w*_11_^(1)^, *w*_12_^(1)^, *w*_13_^(1)^}, {*w*_21_^(1)^, *w*_22_^(1)^, *w*_23_^(1)^}, {*w*_31_^(1)^, *w*_32_^(1)^, *w*_33_^(1)^}, and the bias value is {*b*_1_^(1)^, *b*_2_^(1)^, *b*_3_^(1)^}. The hidden layer has 3 output values {*c*_1_^(2)^, *c*_2_^(2)^, *c*_3_^(2)^}, the weight corresponding to the output layer is {*w*_11_^(2)^, *w*_12_^(2)^, *w*_13_^(2)^}, and the bias value is *b*_1_^(2)^. The output result is represented by *Z*, *f*(*h*) represents the activation function, and the mathematical formula to express this neural network is

(6) $$\begin{array}{c} \left\{\begin{array}{c} c_{1}^{\left(2\right)}=f\left(w_{11}^{\left(1\right)}x_{1}+w_{12}^{\left(1\right)}x_{2}+w_{13}^{\left(1\right)}x_{3}+b_{1}^{\left(1\right)}\right),\\ c_{2}^{\left(2\right)}=f\left(w_{21}^{\left(1\right)}x_{1}+w_{22}^{\left(1\right)}x_{2}+w_{23}^{\left(1\right)}x_{3}+b_{2}^{\left(1\right)}\right),\\ c_{3}^{\left(2\right)}=f\left(w_{31}^{\left(1\right)}x_{1}+w_{32}^{\left(1\right)}x_{2}+w_{33}^{\left(1\right)}x_{3}+b_{3}^{\left(1\right)}\right),\\ Z=f\left(w_{11}^{\left(2\right)}c_{1}^{\left(2\right)}+w_{12}^{\left(2\right)}c_{2}^{\left(2\right)}+w_{13}^{\left(2\right)}c_{3}^{\left(2\right)}+b_{1}^{\left(2\right)}\right). \end{array}\right. \end{array}$$

In the same way, the calculation steps of extending this model to a neural network with *l* layers are roughly similar. Taking *c*_*i*_^*l*^ to represent the output value of the *i* neuron of the *l* layer and *w*_*ij*_^(*l* − 1)^ and *b*_*i*_^(*l* − 1)^ the weight and bias values of the corresponding layer, then formula (7) can be obtained:

(7) $$\begin{array}{c} \left\{\begin{array}{c} h_{i}^{l}=\overset{n}{\underset{j=1}{\sum }}w_{ij}^{\left(l-1\right)}x_{j}+b_{i}^{\left(l-1\right)},\\ c_{i}^{l}=f\left(h_{i}^{l}\right). \end{array}\right. \end{array}$$

BP networks are typical feedforward neural networks, and there are other radial basis function neural networks. A seemingly complex neural network is actually relatively easy to solve. From the first single neuron to two-layer, three-layer, and even multilayer neural networks, you can quickly find the output of your neuron as long as you master the solution, matrix the parameters, and use the fast computing power of your computer.

The article "Correlation between Vaginal Microecological Status and Prognosis of CIN Patients with High-Risk HPV Infection" was published in 2022. Journal: Biomed Res Int.

#### 2.2.3. Reverse Conduction Algorithm

The reverse conduction algorithm can continuously optimize the connection weights and biases between each artificial neuron according to the expected output information; that is, the algorithm can propagate the difference between the expected value and the network output to the input layer layer-by-layer, to modify the weight of the connection. When the error signal is transmitted back to a certain layer, the signal will be allocated to the processing unit of this layer as the basis for modifying the weight of the unit. Backpropagation will continue until the number of iterations or learning times set by the network, or the output error is reduced to the range that the network designer can accept [23–26]. The reverse conduction algorithm is an important part of the neural network. The input layer contains two neurons *x*_1_, *x*_2_ with a bias of *b*_1_; the hidden layer contains two neurons *c*_1_, *c*_2_ with a bias of *b*_2_; the output layer has two values *z*_1_, *z*_2_. There is a weight *w*_*i*_ between each neuron; let the activation function be *f*(*h*). Suppose the total error is *E*, the error of *z*_*i*_ is *e*_*i*_, and the expected output is *t*_*i*_. Then the total error can be obtained by

(8) $$\begin{array}{c} \left\{\begin{array}{c} e_{1}=\frac{1}{2}{\left(t_{1}-z_{1}\right)}^{2},\\ e_{2}=\frac{1}{2}{\left(t_{2}-z_{2}\right)}^{2},\\ E=\left(e_{1}+e_{2}\right)=\sum \frac{1}{2}{\left(t_{i}-z_{i}\right)}^{2}. \end{array}\right. \end{array}$$

Regarding the update of the weight from the hidden layer to the output layer, the *w*_5_ weight in the network can be used for illustration. The calculation formula is shown in Equation (9), and the partial derivative of the total error to *w*_5_ can be obtained:

(9) $$\begin{array}{c} \left\{\begin{array}{c} h_{5}=w_{5}*c_{1}+w_{6}*c_{2}+b_{2}*1,\\ \frac{\partial E}{\partial w_{5}}=\frac{\partial E}{\partial z_{1}}*\frac{\partial z_{1}}{\partial h_{5}}*\frac{\partial h_{5}}{\partial w_{5}}. \end{array}\right. \end{array}$$

Bringing Equation (8) into Equation (9) can get

(10) $$\begin{array}{c} \left\{\begin{array}{c} h_{1}=w_{1}*x_{1}+w_{2}*x_{2}+b_{1}*1,\\ \frac{\partial E}{\partial w_{5}}=-\left(t_{1}-z_{1}\right)*z_{1}\left(1-z_{1}\right)*f\left(h_{1}\right). \end{array}\right. \end{array}$$

Let *η* be the learning rate, the updated value of weight *w*_5_ can be obtained, expressed as *gw*_5_, and the formula is shown in

(11) $$\begin{array}{c} {gw}_{5}=w_{5}-\eta *\frac{\partial E}{\partial w_{5}}. \end{array}$$

For the weight update from the hidden layer to the hidden layer, the errors of *e*_1_ and *e*_2_ must be counted, because the neurons of the hidden layer are fully connected with the output layer. The following takes the weight update of *w*_1_ for explanation. Before calculating the influence of *w*_1_ on the total error *E*, the partial derivatives of *e*_1_ and *e*_2_ with respect to *w*_1_ need to be calculated separately, as shown in

(12) $$\begin{array}{c} \left\{\begin{array}{c} \frac{\partial E}{\partial f\left(h_{1}\right)}=\frac{\partial e_{1}}{\partial f\left(h_{1}\right)}+\frac{\partial e_{2}}{\partial f\left(h_{1}\right)},\\ \frac{\partial E}{\partial w_{1}}=\frac{\partial E}{\partial f\left(h_{1}\right)}*\frac{\partial f\left(h_{1}\right)}{\partial h_{1}}*\frac{\partial h_{1}}{\partial w_{1}},\\ \frac{\partial E}{\partial w_{1}}=\left(\frac{\partial e_{1}}{\partial f\left(h_{1}\right)}+\frac{\partial e_{2}}{\partial f\left(h_{1}\right)}\right)*\frac{\partial f\left(h_{1}\right)}{\partial h_{1}}*\frac{\partial h_{1}}{\partial w_{1}}. \end{array}\right. \end{array}$$

Finally, from Equations (12) and (11), the updated weight of *w*_1_ can be obtained, expressed as *gw*_1_, and the equation is shown in

(13) $$\begin{array}{c} {gw}_{1}=w_{1}-\eta *\frac{\partial E}{\partial w_{1}}. \end{array}$$

By analogy, the update method of other weights *w*_2_, *w*_3_, *w*_4_ is similar. Since then, according to the chain calculation rule, the partial derivatives of weights *w*_1_ and *b*_1_ are calculated as shown in

(14) $$\begin{array}{c} \left\{\begin{array}{c} \delta_{i}^{\left(l\right)}=\left(\overset{S_{l+1}}{\underset{j=1}{\sum }}w_{ij}^{\left(l\right)}\delta_{j}^{\left(l+1\right)}\right)f^{\prime }\left(h_{i}^{\left(l\right)}\right),\\ \frac{\partial J\left(w,b,x,y\right)}{\partial w_{ij}^{\left(l\right)}}=c_{j}^{\left(l\right)}\delta_{i}^{\left(l+1\right)},\\ \frac{\partial J\left(w,b,x,y\right)}{\partial b_{i}^{\left(l\right)}}=\delta_{i}^{\left(l+1\right)}. \end{array}\right. \end{array}$$

Among them, (*w*, *b*) is the weight parameter of the neural network, (*x*, *y*) represents the data set {(*x*^(1)^, *y*^(2)^) ⋯ (*x*^(*m*)^, *y*^(*m*)^)} to be trained by the network and contains *m* training samples, *J*(*w*, *b*, *x*, *y*) is the corresponding loss function of a single training sample (*x*, *y*), and *δ*_*i*_^(*l* + 1)^ is the error of the *i* neural processing unit of the *l* + 1 layer. The reverse conduction algorithm can be summarized as the following: first, calculate the activation value of all neural processing units in each layer of the feedforward transmission process, then calculate the error value of the output results and samples of the network, and then return to the hidden layer to find the error of each node value, and finally, calculate the partial derivative value of the weight. In this way, the calculation method of reverse conduction is completed, and the weights are continuously updated after continuous iteration, so that the output result of the network and the expected value are constantly approaching.

The article "Correlation between Vaginal Microecological Status and Prognosis of CIN Patients with High-Risk HPV Infection" was published in 2022. Journal: Biomed Res Int.

## 3. Experimental Design of the Correlation between Vaginal Microecological Status and Prognosis of CIN Patients

### 3.1. Test Subject

#### 3.1.1. Inclusion Criteria

The case selection criteria were married women who attended a gynecological outpatient clinic of a hospital from January 2020 to September 2021 and had abnormal cervical cancer and precancerous lesion screening. All patients underwent high-risk HPV testing and vaginal microbiology with informed consent and ecological testing.

#### 3.1.2. Elimination Criteria

The elimination criteria are the following: incomplete case data, being treated with immunosuppressive agents, vaginal washing and medication 3 days before specimen collection, and a history of high-risk HPV infection in the past, who turned negative during this examination.

#### 3.1.3. Grouping Standard

There are 280 cases in the experimental group: the first high-risk HPV test results were found to be positive 6 months ago; this time, the high-risk HPV test was still positive. There are 140 cases in the control group: all were healthy people, and no high-risk HPV infection was found before. The second-high-risk HPV test was negative. Follow-up was performed 3, 6, 9, 12, 18, and 24 months after standard treatment. Among them, 240 high-risk HPV-positive patients underwent regular cytology and high-risk HPV testing until they turned negative. The results of vaginal microecological testing and high-risk HPV load and cervical lesions of various grades were analyzed.

The article "Correlation between Vaginal Microecological Status and Prognosis of CIN Patients with High-Risk HPV Infection" was published in 2022. Journal: Biomed Res Int.

### 3.2. Method of Obtaining Vaginal Secretions

Candidates lie on the gynecological examination table and take the bladder lithotomy position; the sterilized speculum was lubricated with a small amount of sterilized normal physiological saline and placed in the candidate's vagina to completely expose the cervix. And in particular, during the vaginal microecological examination, use a sterile cotton swab to remove vaginal secretions from the upper third of the vaginal sidewall, rotate the cotton swab, and stay on the vaginal sidewall for 15-20 seconds. After the swab is completely immersed in the specimen, carefully place it in a dry, sterile test tube and avoid contact with the vagina or vulva during this period to prevent contamination of the specimen. Then gently insert the high-risk HPV sample collection brush into the cervix and rotate the sample collection brush 5 times clockwise. After brushing enough cervical epithelial cells, carefully place the specimen sampling brush on the high-risk specimen. A special sterile sampling tube used for HPV storage reagents breaks the brush handle and closes the mouth of the sampling tube tightly. During this period, avoid touching the vagina or vulva to prevent contamination of the specimen. The above samples were collected by two obstetricians and a gynecologist and sent to the laboratory for examination by a professional inspector within 1 hour of the sample being taken. Professional inspectors strictly follow the operating procedures of the bPR-2014A Vaginal Microecological Evaluation System for cytological and functional examination of vaginal discharge.

### 3.3. High-Risk HPV Detection and Criteria

For the standard high-risk HPV test result determination, the content of high-risk HPV is determined by the ratio of relative light unit to the standard positive control, relative light unit/standard positive control < 1 is judged as negative, relative light unit/standard positive control ≥ 1 is judged as positive, and the larger the relative light unit/standard positive control value, the higher the load value of the high-risk HPV virus.

### 3.4. Follow-Up Method

With informed consent of all patients, the knowledge about cervical cancer and its precancerous lesions shall be promoted and popularized one by one, and basic information such as the patient's name, age, contact number, home address, pregnancy times, parity, and interroom bleeding shall be collected. The pathological diagnosis of biopsy means that standard treatment is given, and patients are instructed to strictly follow the doctor's instructions. Follow-ups will be conducted at 3, 6, 9, 12, 18, and 24 months after treatment. Cervical cytology and high-risk HPV testing will be performed at each follow-up. If necessary, a biopsy can be taken again.

The article "Correlation between Vaginal Microecological Status and Prognosis of CIN Patients with High-Risk HPV Infection" was published in 2022. Journal: Biomed Res Int.

### 3.5. Statistical Processing

Statistical analysis was performed with SPSS 13.0 statistical software. The significance test of the difference was performed by one-way analysis of variance. The difference between the two groups was performed by the LSD *t*-test. The statistics of the vaginal microecological status of CIN patients with high-risk HPV infection were performed by a group *t*-test. *P* < 0.05 is considered to be significant and statistically significant.

## 4. Experimental Correlation between Vaginal Microecological Status and Prognosis of CIN Patients

### 4.1. Morphological Test Results of Vaginal Microecology in Experimental Group and Control Group

#### 4.1.1. Test Results of Vaginal Cluster Density

The 280 cases of the experimental group and 140 cases of the control group were tested for the concentration of vaginal clusters. The results are shown in Figure 2.

It can be seen from Figure 2 that the concentration of vaginal secretion flora between 0 and I indicates that the flora is inhibited. The detection rate of vaginal secretion flora in the experimental group between 0 and I is 2.50% (7/280); the detection rate of the control group was 2.14% (3/140). Compared with the two, the detection rate of vaginal flora suppression in the experimental group was lower than that of the control group. The density of normal vaginal microecological flora should be between II and III, the detection rate of the experimental group's flora density is between II and III 96.43% (270/280), and the detection rate of the control group is 97.86% (137/140). Comparing the two, the normal rate of vaginal flora density in the experimental group was lower than that in the control group. Vaginal flora density grade IV indicates the excessive proliferation of vaginal flora. The detection rate of bacterial flora density grade IV in the experimental group was 1.07% (3/280), and the detection rate in the control group was 0. Comparing the two, the experiment detection rate of vaginal flora hyperproliferation in the group was higher than that in the control group. There was no statistically significant difference in the overall composition of the two groups (*χ*^2^ = 2.733, *P* > 0.05).

The article "Correlation between Vaginal Microecological Status and Prognosis of CIN Patients with High-Risk HPV Infection" was published in 2022. Journal: Biomed Res Int.

#### 4.1.2. Test Results of Vaginal Flora Diversity

The 280 cases of the experimental group and 140 cases of the control group were tested for the diversity of vaginal flora. The results are shown in Figure 3.

It can be seen from Figure 3 that the density of vaginal flora between 0 and I indicates that the diversity of flora is reduced, and the detection rate of the experimental group's flora diversity between 0 and I is 6.07% (17/280). The detection rate of the control group was 4.29% (6/140); comparing the two, the detection rate of decreased vaginal flora diversity in the experimental group was higher than that in the control group. The diversity of the normal vaginal microecological flora should be between II and III. The detection rate of the experimental group's flora diversity is between II and III 92.86% (260/280), and the detection rate of the control group is 95.71% (134/140). Comparing the two, the normal rate of vaginal flora diversity in the experimental group was lower than that in the control group. The level of vaginal flora diversity indicates that the diversity of flora is too high. The detection rate of level IV of the experimental group's flora diversity is 1.07% (3/280), and the detection rate of the control group is 0. Comparing the two, the detection rate of excessive vaginal flora in the experimental group was higher than that in the control group. There was no statistically significant difference in the overall composition ratio between the two groups (*χ*^2^ = 1.176, *P* > 0.05).

#### 4.1.3. Test Results of Dominant Vaginal Bacteria

280 cases of the experimental group and 140 cases of the control group were tested for vaginal dominant bacteria; the results are shown in Figure 4.

It can be seen from Figure 4 that nondominant bacteria represent the inhibition of vaginal flora. The detection rate of nondominant bacteria in the vaginal flora in the experimental group was 2.14% (6/280), and the detection rate in the control group was 1.43% (2/140). Comparing the two, the detection rate of bacterial colony inhibition in the experimental group has a rising trend, and the difference is not statistically significant. The dominant bacteria in healthy vaginal microecology are Lactobacillus, which is Gram-positive bacteria; the detection rate of Gram-positive bacteria in the experimental group is 74.64% (209/280), and the detection rate in the control group is 90.0% (126/140). Comparing the two, the normal detection rate of dominant bacteria in the experimental group has a decreasing trend. The detection rate of the non-Gram-positive large bacterium as the dominant bacteria in the experimental group was 23.21% (65/280), and the detection rate in the control group was 8.57% (12/140); comparing the two, the detection rate of the dominant bacteria in the experimental group was out of balance; the rate has an upward trend. There was no statistically significant difference in the overall composition ratio between the two groups (*χ*^2^ = 0.62, *P* > 0.05).

The article "Correlation between Vaginal Microecological Status and Prognosis of CIN Patients with High-Risk HPV Infection" was published in 2022. Journal: Biomed Res Int.

#### 4.1.4. Vaginal Secretion White Blood Cell Count/High-Powered Visual Field Results

280 cases of the experimental group and 140 cases of the control group were tested for vaginal secretion white blood cell count. The results are shown in Table 1.

It can be seen from Table 1 that the number of white blood cells in normal vaginal secretions is ≤10/high-power field, and the white blood cell count > 10/high-power field indicates that there may be vaginal inflammation. In the experimental group, the detection rate of vaginal secretion white blood cell count > 10/high-powered visual field was 34.64% (97/280). In the control group, the detection rate of vaginal secretion white blood cell count > 10/high-powered visual field was 39.29% (55/140); comparing the two, the detection rate of inflammation in the experimental group was higher than that in the control group. Calculating the comparison of the overall composition of the two groups, the difference between the two was not statistically significant (*χ*^2^ = 0.004, *P* > 0.05).

#### 4.1.5. Measurement Results of Vaginal pH

The 280 cases of the experimental group and 140 cases of the control group were tested for vaginal pH. The results are shown in Table 2.

It can be seen from Table 2 that the normal vaginal pH value is between 3.8 and 4.5, and the pH value is higher than 4.6 abnormally. The detection rate of pH value > 4.6 in the experimental group was 88.93% (249/280), and the detection rate in the control group was 73.57% (103/140). Compared with the control group, the detection rate of pH value > 4.6 in the experimental group has a rising trend, and the difference in the overall composition ratio between the two groups is statistically significant (*χ*^2^ = 5.372, *P* < 0.05).

#### 4.1.6. Test Results of Vaginal Microecological Enzymes

280 cases of the experimental group and 140 cases of the control group were tested for vaginal microecological enzymes. The results are shown in Table 3.

Table 3 shows that the normal detection rate of hydrogen peroxide in vaginal discharge in the experimental group was 66.43% (186/280), and the detection rate in the control group was 76.43% (107/40). The normal detection rate of hydrogen peroxide in secretions tends to decrease, and the difference is statistically significant (*χ*^2^ = 5.182, *P* < 0.05). The detection rate of sialidase positive in the vaginal discharge of the experimental group was 29.29% (82/280), while the detection rate of the control group was 14.29% (20/140), and the difference was statistically significant. It was *χ*^2^ = 8.233, *P* < 0.05. The detection rate of positive leukocyte esterase in vaginal discharge in the experimental group was 71.79% (201/280) compared to the detection rate of 55.0% (77/140) in the control group, and the difference was statistically significant (*χ*^2^ = 9.349, *P* < 0.05). Compared with the control group, the vaginal discharge in the experimental group had a higher detection rate of *β*-glucuronidase and acetylglucosaminidase, but the difference was not statistically significant.

The article "Correlation between Vaginal Microecological Status and Prognosis of CIN Patients with High-Risk HPV Infection" was published in 2022. Journal: Biomed Res Int.

#### 4.1.7. Comprehensive Evaluation Results of Vaginal Microecological Status

The 280 cases of the experimental group and 140 cases of the control group were comprehensively evaluated for the vaginal microecological status, and the results are shown in Figure 5 and 6.

It can be seen from Figure 5 that the detection rate of normal vaginal microecology in the experimental group was 12.14% (34/280) compared with the detection rate of 29.29% (41/140) in the control group, and the difference was statistically significant (significance (*χ*^2^ = 17.23, *P* < 0.05)). The detection rate of vaginal BV in the experimental group was 10.36% (29/280) compared with the detection rate of 5.0% (7/140) in the control group, and the difference was statistically significant (*χ*^2^ = 5.19, *P* < 0.05). The detection rate of VVC, TV, vaginal flora abnormality, and dysfunction in the experimental group was higher than that of the corresponding control group, but the difference was not statistically significant.

### 4.2. Relevant Results for Patient Prognosis

The age composition of cervical lesions of each grade is different. Therefore, by comparing the relationship between high-risk HPV and cervical lesions of each grade, the age factor should be controlled. The 280 high-risk HPV-positive patients were divided into three groups: ≤35 years old, 36 years old~, and >50 years old. The results are shown in Table 4.

It can be seen from Table 4 that, stratified by age, the high-risk HPV load of each level of cervical lesions was compared by the rank sum test of multiple samples, and the differences were statistically significant (*P* < 0.05). It shows that there are significant differences in the high-risk HPV load of different grades of cervical lesions. And as the level of cervical lesions increases, the load of high-risk HPV also increases significantly. In addition, in patients with chronic cervicitis, CINII~III, and cervical cancer, there was no significant difference in the high-risk HPV load of each age group (*P* > 0.05), indicating that there is no correlation between age and high-risk HPV load. Only in CINI patients, there was a statistically significant difference in the load of high-risk HPV in each age group (*P* < 0.05). With the increase of age, the load of high-risk HPV decreased.

The article "Correlation between Vaginal Microecological Status and Prognosis of CIN Patients with High-Risk HPV Infection" was published in 2022. Journal: Biomed Res Int.

In the chronic cervicitis group, 45.4% of high-risk HPV cases were negative, and the remaining 54.5% of high-risk HPV-positive cases were 34.5%, 10.7%, and 9.4%, respectively. In the CINI group, 28.0% of cases were high-risk HPV-negative, and 72.0% of high-risk HPV-positive cases were 28.4%, 24.3%, and 19.3%, respectively. 7.7% of CINII-III cases were high-risk HPV-negative, and 92.3% of high-risk HPV-positive cases were 30.0%, 40.5%, and 21.8 with low-, moderate-, and high-level loads, respectively. In the cervical cancer group, 4.1% of cases were high-risk HPV-negative, and 95.9% of high-risk HPV-positive cases were 27.5%, 41.9%, and 26.5%, respectively. The load distribution of high-risk HPV in each grade of cervical lesions was compared by multiple sample rate *χ*^2^ tests, and the difference was statistically significant (*χ*^2^ = 231.119, *P* < 0.05). This indicates that the high-risk HPV infection rates for different grades of cervical lesions differ significantly and that the high-risk HPV infection rates increase significantly with the level of cervical lesions.

## 5. Conclusions

Multiple HPV infections can increase the risk of cervical lesions. On the one hand, it may be related to the interaction between HPV subtypes. On the other hand, more and more reports about HPV recombination suggest that multiple HPV infections may increase the risk of HPV recombination, producing HPV that is carcinogenic. This article analyzes the correlation between the vaginal microecological status of high-risk HPV-infected CIN patients and the patients' prognosis. Compared with healthy women, women with high-risk HPV infection for more than 6 months have the vaginal flora density of women with high-risk HPV infection for more than 6 months. The detection rates of abnormalities, abnormal flora diversity, dominant bacteria, vaginal secretion white blood cell count > 10/high-powered field of view, and *β*-glucuronidase-positive and acetylglucosaminidase-positive detection rates are all higher than those of the control group. There is no statistical significance (*P* > 0.05). The shortcomings of this article are the following: Because vaginal microecological testing is a new type of testing method, most medical institutions have not introduced the testing equipment, and the patients' acceptance of this testing method is not high, resulting in the failure of this study to be carried out on a large scale and many times. Center clinical trials can lead to inaccurate statistical results. Although there is a certain relationship between changes in female vaginal microecological status and long-term high-risk HPV infection, the specific mechanism remains unclear, and further studies are needed. Functional vaginal microecosystems play an important role in combating high-risk HPV infections. In the future, it will be used to increase the quantity and quality of lactic acid bacteria in the vagina, restore normal levels of hydrogen peroxide, and regulate vaginal pH when diagnosing and treating high-risk HPV infections. I can do it. And methods of killing pathogenic microorganisms improve the cure rate of high-risk HPV infections in many ways.

The article "Correlation between Vaginal Microecological Status and Prognosis of CIN Patients with High-Risk HPV Infection" was published in 2022. Journal: Biomed Res Int.

## Figures and Tables

**Figure 1:** Feedforward neural network structure.

**Figure 2:** The density of vaginal microecological flora in the two groups of research subjects.

**Figure 3:** Diversity of vaginal flora in the two groups of subjects.

**Figure 4:** The status of dominant vaginal bacteria in the two groups of subjects.

**Figure 5:** Comprehensive evaluation of vaginal microecology in the two groups of subjects.

**Figure 6:** Schematic diagram of the distribution of high-risk HPV load of various levels of cervical lesions.

**Table 1:** Vaginal secretion white blood cell count/high-powered visual field of the two groups of research subjects.

White blood cell count	Experiment group		Control group	
	Number of cases	Composition ratio (%)	Number of cases	Composition ratio (%)
≤10	183	65.36	85	60.71
>10	97	34.64	55	39.29

**Table 2:** The measurement of vaginal pH value of the two groups of research subjects.

Vagina pH	Experiment group		Control group	
	Number of cases	Composition ratio (%)	Number of cases	Composition ratio (%)
3.8~4.5	31	11.07	37	26.43
>4.6	249	88.93	103	73.57

**Table 3:** The vaginal microecological enzymes of the two groups of research subjects.

Functional indicators	Experiment group		Control group		*χ* ^2^	*P*
	Number of cases	Composition ratio (%)	Number of cases	Composition ratio (%)		
Hydrogen peroxide is normal	186	66.43	107	76.43	5.182	<0.05
Hydrogen peroxide deficiency	94	33.57	33	23.57		

Sialidase positive	82	29.29	20	14.29	8.233	<0.05
Sialidase negative	198	70.71	120	85.71		

Leukocyte esterase positive	201	71.79	77	55.00	9.349	<0.05
Leukocyte esterase negative	79	28.21	63	45.00		

*β*-Glucuronidase positive	6	2.14	1	0.71	0.325	>0.05
*β*-Glucuronidase negative	274	97.86	139	99.29		

Acetylglucosaminidase positive	14	5.00	6	4.29	0.074	>0.05
Acetylglucosaminidase negative	266	95.00	134	95.71		

The article "Correlation between Vaginal Microecological Status and Prognosis of CIN Patients with High-Risk HPV Infection" was published in 2022. Journal: Biomed Res Int.

**Table 4:** Comparison of HR-HPV load of various cervical lesions.

Year	Chronic cervicitis		CINI		CINII~III		Cervicitis		Statistics	*P*
	*M*	*Q*	*M*	*Q*	*M*	*Q*	*M*	*Q*		
≤35	2.700	0.588	3.450	2.311	8.965	6.968	1.440	3.572	4.200	<0.05
36~	1.173	0.510	7.335	0.783	5.290	8.020	0.398	4.826	14.759	<0.05
>50	1.294	0.460	1.782	0.545	5.525	2.983	6.150	7.938	4.656	<0.05
Statistics	2.411		4.416		1.892		0.436		—	—
*P*	>0.05		<0.05		>0.05		>0.05		—	—

## Data Availability

The data used to support the findings of this study are included within the article.
